# Psychometric properties of a short version of the Job Anxiety Scale

**DOI:** 10.1186/s12874-020-00974-4

**Published:** 2020-04-21

**Authors:** Bjarne Schmalbach, Andreas Kalkbrenner, Markus Bassler, Andreas Hinz, Katja Petrowski

**Affiliations:** 1 Department of Psychosomatic Medicine and Psychotherapy, University Medical Center of the Johannes Gutenberg University Mainz, Untere Zahlbacher Str. 8, 55131 Mainz, Germany; 2 Technische Universität Dresden, University Hospital Carl Gustav Carus, Clinic of Psychotherapy and Psychosomatic Medicine, Fetscherstraße 74, 01307 Dresden, Germany; 3 Hochschule Nordhausen, University of Applied Sciences, Weinberghof 4, 99734 Nordhausen, Germany; 4 Department of Medical Psychology and Medical Sociology, University of Leipzig, Philipp-Rosenthal-Str. 55, 04103 Leipzig, Germany; 5 University Medical Center of the Johannes Gutenberg University Mainz, Medical Psychology and Medical Sociology, Duesbergweg 6, 55131 Mainz, Germany

**Keywords:** Job anxiety scale, JAS, Job related anxiety, Screening instrument, Scale construction, Job assessment, (215 words)

## Abstract

**Background:**

Occupational stress and specifically job anxiety are crucial factors in determining health outcomes, job satisfaction as well as performance. In order to assess this phenomenon, the Job Anxiety Scale is one of the instruments available. It consists of 70 items that are clustered in 14 subscales and five dimensions. The aim of this paper is to create a more efficient, short version of the Job Anxiety Scale, while retaining the five dimensions, and to assess its psychometric properties.

**Methods:**

The sample consists of 991 – mostly psychosomatic – patients from two different clinics. We applied methods of factor analysis and bivariate correlations to explore and test factor structure and the nomological net of related constructs.

**Results:**

After reducing the item pool via the construction of subsets and tests using ant-colony-optimization, a 15-item version of the Job Anxiety Scale evinced very good psychometric properties. We found very good model fit, high internal consistency, and invariance across participant age and sex. It displayed improved discriminant validity compared to the original scale, and we found the expected pattern of convergent correlations.

**Conclusions:**

With this short version of the Job Anxiety Scale, researchers can assess job related worries in a much more economic manner. The questionnaire is particularly useful in large-scale surveys and/or in samples that struggle with extensive assessments.

## Background

Occupational stressors are crucial predictors in explaining a wide range of positive and negative job-related outcomes. For instance, higher levels of job-related stress and anxiety have been shown to be related to lower levels of job satisfaction and commitment to the job [1, 2]. Motowidlo, Packard, and Manning [3] even suggest an impact on performance based on the frequency of stressful experiences. It is estimated that almost 5% of German employees are at risk of being absent from work because of job anxiety [4]. This fact is associated with high costs for companies, health insurance and public pension funds. Thus, research into the phenomenon and a reliable and valid assessment of the construct are of great interest to researchers and practitioners alike.

People who experience job anxiety feel typical anxiety symptoms such as trembling, blushing or palpitations when they are at work or when they think of their work [5]. Even though these symptoms have a major influence on work performance, there is no ICD code for work place phobia. Haines, Williams, and Carson [6] used the criteria of phobia to characterize workplace related anxieties: intense anxiety when approaching the workplace, incapacity to enter the workplace because of anxiety respectively panic symptoms and a reduction of anxiety when leaving the workplace. Bryson, Barth, and Dale-Olsen [7] used parts of Warr’s anxiety-contentment axis model [8] for measuring job anxiety. Even though it is a clinically and economically important construct, there is only one questionnaire available for measuring job anxiety - the Job Anxiety Scale (JAS) [9].

Muschalla [10] ran a pilot study, using an initial version of the JAS with 106 items. This version contained criteria of anxiety related to ICD 10 [11], DSM-IV [12] and patient reported aspects of job related anxieties. Based on this first trial, Linden, Muschalla, and Olbrich [9] modified the scale into its current version containing 70 items. The 70 items of the JAS questionnaire are clustered by theoretical assumptions in 14 subscales and five dimensions. The five dimensions assess issues related to stimulus-related anxiety and avoidance behavior, social anxieties and cognition of mobbing, health- and body-related anxieties, cognitions of insufficiency, as well as job-related worrying. An overview of all JAS dimensions and a selection of items can be found in Table 1. For the assessment of job-related anxiety each subscale and dimension as well as a global mean value can be analyzed based on the 70 JAS items. The psychometric properties of the JAS show very good values for Cronbach’s alpha (α = .98 [9];). The JAS also shows good results for retest-reliability: .85 [9] and .82 [4]. Concerning convergent validity, the correlation with the Stait-Trait Anxiety Inventory (STAI-T [13] resulted in .69 [9] and .67 [4]. Job stressors and anxiety have been shown to be associated positively with adverse mental health outcomes [5, 14], and negatively with social support and well-being [15–17].

**Table 1:** Descriptive statistics of the JAS-15 items and scales

	*M*	*SD*	γ1	γ2	*r*_*it*_	λ	ω
Stimulus-related anxiety and avoidance behavior	1.064	1.152	.962	−.145			.784
Whenever possible, I avoid coming near to the site of my workplace.	.940	1.368	1.221	.050	.671	.800	
After work, I hurry up more than others just to get away from that place.	1.143	1.389	.947	−.469	.638	.794	
I have once experienced a terrible event at the workplace which is still present in my mind and makes me feel frightened at work.	1.110	1.420	1.016	−.398	.505	.627	
Social anxiety and cognition of mobbing	1.072	1.084	.913	−.071			.745
At the workplace, I have got problems with one or more colleagues.	.994	1.233	1.229	.470	.540	.568	
I have got problems with one or more superiors.	1.238	1.439	.883	−.640	.611	.688	
At my workplace I am in the mercy of persons´ arbitrary behaviors and unfairness.	.985	1.278	1.192	.261	.628	.836	
Health- and body-related anxieties	1.619	1.324	.440	−1.084			.921
My work ruins my state of health.	1.572	1.408	.492	−1.065	.687	.924	
If I stay any longer at this workplace, this will cause harm to my health.	1.548	1.463	.527	−1.120	.843	.889	
The stress at my workplace is causing ill health.	1.737	1.413	.335	−1.181	.796	.860	
Cognition of insufficiency	1.690	1.226	.315	−1.054			.825
The conditions under which I work make me nervous.	1.654	1.405	.382	−1.148	.743	.884	
I have miserable feelings at my workplace which restrict my capacities for achievement.	1.828	1.406	.230	−1.266	.682	.735	
I suffer from the fact that I never know what comes up next at my workplace.	1.587	1.429	.451	−1.160	.667	.722	
Job-related worrying	1.653	1.225	.334	−.991			.854
I am always worrying about minor matters in my work and during all the working day.	1.734	1.365	.342	−1.110	.789	.910	
Colleagues or family have already told me that I should not always worry that much about work.	1.491	1.399	.538	−1.006	.547	.594	
I am suffering from the worries which I cannot put away or stop.	1.735	1.470	.308	−1.296	.771	.907	
JAS Total Score	1.420	1.031	.538	−.669			.953

*M* = Mean; *SD* = Standard deviation; γ1 = skewness; γ2 = excess kurtosis; *r*_*it*_ = corrected item-total correlation for the shortened scales; λ = standardized factor loading; ω = reliability coefficient

For a more economical way of screening job related anxiety there is a Workplace Phobia Scale (WPS [18]). This questionnaire consists of 13 out of the 70 items. These items were selected from the JAS – not empirically driven. The authors took all items from the subscales Anticipatory anxiety (five items), Phobic avoidance (six items) and the two items of the Global workplace-anxiety subscale. Since anticipatory anxieties and avoidance behavior are the central aspects of phobia, the WPS captures phobia and criteria of clinic disorders.

However, the WPS does not allow to capture a wide non-phobia, clinic-specific, comprehensive assessment of job anxieties in the manner the JAS does. Specifically, cognitions of mobbing and insufficiency as well as health-related thought patterns are not captured. We seek to remedy this issue with the present study. Furthermore, as job anxiety is not an ICD diagnoses or clinical diagnoses, there is a need for a scale, which measures work-related worries as a wider construct but in a more economic manner. Especially for big surveys in non-clinical and work-related contexts a shorter version to measure job anxieties needs to be established. Therefore, the aim of this study is to create an empirically derived, economic, short version of the JAS and the assessment of its psychometric properties. To this end, we will reduce the initial 70-item JAS by statistical means while retaining the five theoretically meaningful dimensions. To allow for the construction of an efficient screening instrument, we aim to retain three items per dimension. In addition, we will investigate the shortened scales with regard to their convergent validity by examining its associations with a measure of psychosocial health.

## Methods

### Study sample

We recruited the sample in the Clinic of Psychotherapy and Psychosomatic Medicine, University Hospital Dresden (*n* = 284) and the Rehabilitation Center Oberharz (*n* = 758). We focused on patients and individuals in rehabilitation because, first, the JAS was developed in a similar setting [9], and second, such as sample (vs. a general population sample) will yield a broader distribution of the characteristic in question.

Description Dresden: Included are 169 females (59.5%) with a mean age of 36.64 (*SD* = 13.19) years and 115 males (40.5%) with a mean age of 37.39 (*SD* = 12.20) years. The overall mean age of the sample was 36.94 (*SD* = 12.88; range, 17 to 83) years. 26.7% of the sample lived alone in their household, 71.5% of the sample lived together with one or more people. The diagnoses for this group are displayed in Table 2.

**Table 2:** Diagnoses of both subsamples

*Diagnoses of the Patients from the Technische Universität Dresden, University Hospital Carl Gustav Carus (n = 277)*		
	Frequency	%
F40–48 - Neurotic, stress-related and somatoform disorders	151	54.5
F30–39 - Mood (affective) disorders	89	32.1
F50–59 - Behavioural syndromes associated with physiological disturbances and physical factors	4	1.4
F10–19 - Mental and behavioural disorders due to psychoactive substance use	3	1.1
Other diagnoses	30	10.8
*Diagnoses of the Inpatients from the Rehabilitation Center Oberharz (n = 758)*		
	Frequency	%
F40–48 - Neurotic, stress-related and somatoform disorders	387	51.1
F30–39 - Mood (affective) disorders	304	40.1
M50–54 - Other dorsopathies	35	4.6
F60–69 - Disorders of adult personality and behaviour	8	1.1
Other diagnoses	24	3.2

Description Oberharz: The second group (*N* = 758) consists of patients from the “Rehabilitation Center Oberharz” (Rehazentrum Oberharz). Four hundred eleven females (54.2%) with a mean age of 46.90 (*SD* = 8.66) years and 347 males (45.8%) with a mean age of 47.14 (*SD* = 9.99) years were assessed in this sample. The overall mean age of the sample was 47.01 (*SD* = 9.29; range, 18 to 74) years. The diagnoses for this group are also displayed in Table 2.

All participants volunteered and received a data protection declaration in agreement with the Helsinki Declaration. The study was approved the ethics committee of the Medical Faculty of the Technische Universität, Dresden (EK 79032011). Verbal and written informed consent was obtained from all participants.

The JAS questionnaire [9] has already been described in the section “Background.” It consists of five dimensions, 14 subscales and 70 items. Each item was scored on a 5-point Likert scale, ranging from of 0 (no agreement) to 4 (full agreement) – with no reverse-scored items. Reliability (Cronbach’s α) was reported as being .96 [9].

We used the Hamburg Modules for the Assessment of Psychosoical Health (HEALTH [19, 20]) to measure general psychosocial well-being and health in the respondents. It uses 49 items to assess nine subscales (and a psychological symptoms aggregate), which include among others mental health symptoms, self-efficacy, well-being, as well as social support and participation. As per Rabung et al. [19], internal consistency is acceptable to very good for all subscales with values between α = .73 and .91.

### Statistical analyses

All analyses were performed in R, using the packages *lavaan*, *lordif semTools*, and *stuart* [21–24]. Missing values were replaced by linear interpolation up to a limit of 5% missing values. Data sets containing more than 5% missing values were deleted. In accordance with Hair, Black, Babin, and Anderson [25] and Kim [26], we first eliminated those items that evinced unacceptable descriptive statistics with regard to their item-total correlation (*r*_*it*_ < .50), their skewness (> |2|), and their excess kurtosis (> |4|).

Next, we randomly split the full sample (*n* = 991) into an exploratory (*n* = 489) and a confirmatory subsample (*n* = 502). Using the exploratory sample, we further reduced the remaining item pool of 64 items to 15 items (five scales, three items per scale). *Stuart* employs ant-colony-optimization to construct and test subsets of the given indicators for a given factor structure. Apart from a 5 factor × 3 item structure, we constrained the algorithm to prefer solutions that are strongly invariant across participant sex. We then conducted confirmatory factor analysis using *lavaan* in the confirmatory subsample, using robust maximum likelihood estimation [27] and robust formulas for the estimation of fit indices [28, 29]. To evaluate model fit, we employed the commonly recommended indicators and cutoffs [30, 31]: χ^2^-test (non-significant), χ^2^/*df* (< 2), Comparative Fit Index (*CFI* > .95), the Tucker-Lewis Index (*TLI > .95*), the Root Mean Square Error of Approximation (*RMSEA* < .08), and the Standardized Root Mean Square Residual (*SRMR* < .08). We report reliability as McDonald’s ω, which is the preferred measure of internal consistency [32].

For the investigation of measurement invariance, we used the common step-wise model comparison approach [33]. In this procedure, one compares increasingly restrictive models to establish increasingly strict levels of invariance. Specifically, the first step is the comparison of the configural (unconstrained) model with the metric (equal factor loadings across compared groups) model. Second, one compares the metric to the scalar (equal item intercepts across compared groups) model. Finally, one compares the scalar to the strict (equal residual terms across compared groups) model. To evince measurement invariance, χ^2^ should not be significant and the difference in *CFI* and gamma hat (*GH*) should not exceed .01 [34].

To supplement these analyses, we conducted analyses of differential item functioning (DIF) using the *lordif* package [21]. *lordif* is based in the item response theory framework and utilizes ordinal logistic regression to compare models that account for the effects of (1) ability, (2) ability + group, and (3) ability + group + the ability-X-group interaction. Differences between Models 1 and 2 represent the influence of uniform DIF (which corresponds to group-specific item intercepts in the factor analysis framework), whereas differences between Models 2 and 3 represent the influence of non-uniform DIF across the trait spectrum (which corresponds to differences in factor loadings).

## Results

Descriptive statistics were satisfactory for most of the JAS items. Only six items failed the standards with regard to their item-total correlation (24, 31, 70, 53) and their skewness (52, 56) and were removed from consideration. The remaining 64 items were then input into *stuart* for exploratory analysis. Among the 7.56 × 10^11^ possible combinations, the algorithm revealed the best model fit for the items displayed in Table 1, χ^2^(185) = 218.347, *p* = .047, χ^2^/*df* = 1.180, *CFI* = .994, *TLI* = .993, *RMSEA* (90% *CI*) = .027 (.003; .041), *SRMR* = .039. Next, we tested the discovered model structure in the independent confirmatory sample, which again revealed very good fit, χ^2^(80) = 171.046, *p* < .001, χ^2^/*df* = 1.629, *CFI* = .980, *TLI* = .974, *RMSEA* (90% *CI*) = .048 (.039; .056), *SRMR* = .036, affirming the reduced model. Factor loadings exceeded .50 for all indicators (.568 ≤ λ ≤ .924), and reliability coefficients were between ω = .745 and .921 for the five subscales and ω = .953 for the total score (see Table 1). The shortened JAS-15 total score correlates very highly with the JAS-70, *r* = .973, *p* < .001. To further compare the long and short forms of the JAS, we generated test information curves for both versions. As can be seen in Fig. 1, both scales have similar distributions that can be considered reasonably precise from about -2θ to +2θ. It should be noted, that the JAS-15 (vs. the JAS-70) has an information distribution that is more closely centered around the average trait value of 0. This means that it assesses more evenly across the trait spectrum, unlike the JAS-70, which has a more pronounced left-skew.

**Fig. 1:** Test information functions for JAS-70 and JAS-15. JAS = Job Anxiety Scale

In order to justify the computation of a total score, we also tested a second-order factor model, in which all of the subscales loaded onto a second-order latent variable. This model only decreased marginally in terms of its fit, χ^2^(85) = 257.693, *p* < .001, χ^2^/*df* = 3.032, *CFI* = .977, *TLI* = .971, *RMSEA* (90% *CI*) = .053 (.046; .061), *SRMR* = .036. A substantial amount of total variation is explained by the second-order factor, ω_L1_ = .909. This result confirms the validity of the total scale score. However, this should not be taken as a sign for the redundancy of the subfactors: A unidimensional model attains unacceptable fit, χ^2^(90) = 1026.056, *p* < .001, χ^2^/*df* = 11.401, *CFI* = .868, *TLI* = .846, *RMSEA* (90% *CI*) = .123 (.116; .130), *SRMR* = .055, despite its very high internal consistency of ω = .942.

We then tested the measurement invariance of the 5-factor model across participant sex and age. To avoid statistical dependence with the exploratory analyses, we used only the confirmatory sample when investigating invariance across sex. The results of these analyses are reported in Table 3. There is clear evidence for strict invariance across both sex and age groups. The χ^2^-difference test was (marginally) significant for only one of the six model comparisons, and neither Δ*CFI* nor Δ*GH* exceed .01 between specifications.

**Table 3:** Fit indices for the analysis of measurement invariance

Model	χ^2^(*df*)	Δχ^2^	Δ*df*	Δ*p*	*CFI*	Δ*CFI*	*GH*	Δ*GH*
Sex								
Female	156.813 (85)				.978		.978	
Male	166.236 (85)				.980		.981	
Multigroup analysis								
Configural invariance	301.099 (170)				.965		.966	
Metric invariance	325.179 (184)	24.081	14	.045	.963	.002	.964	.002
Scalar invariance	340.284 (193)	15.104	9	.088	.962	.001	.962	.002
Strict invariance	348.501 (208)	8.218	15	.915	.963	.001	.964	.002
Age, years								
≤ 40	140.098 (85)				.976		.978	
41–50	164.961 (85)				.966		.968	
≥ 51	131.966 (85)				.984		.982	
Multigroup analysis								
Configural invariance	437.914 (255)				.976		.976	
Metric invariance	466.423 (283)	28.508	28	.438	.976	.000	.976	.000
Scalar invariance	493.446 (301)	27.023	18	.079	.975	.001	.975	.001
Strict invariance	528.328 (331)	34.882	30	.247	.974	.001	.974	.001

χ^2^ = scaled chi square statistic; *CFI* = robust comparative fit index; GH = scaled gamma hat. For participant sex, the analysis was only conducted in the confirmatory sample to avoid statistical dependence with the exploratory analysis

To supplement these findings, we conducted item-specific comparisons in *lordif*.

In terms of participant sex, we observed a significant χ^2^-test (*p* < .001) for Item 10 with regard to non-uniform DIF. However, the *Pseudo R*^*2*^_*Nagelkerke*_ indicated only a very small effect size. With regard to participant age, we again found a significant χ^2^ between groups for Item 10 (*p* < .001), but also for Item 7 (*p* < .001). This time the effects indicated uniform DIF, yet the effect sizes were again negligibly small: *R*^*2*^_*Nagelkerke*_ *=* .006 and .003, respectively.

Thus, the analysis of DIF and the multigroup confirmatory factor analysis overall yielded the same result: There is no substantial influence of sex or age on the measurement processes of the JAS-15.

Next, we examined the convergent validity of the JAS-15 (see Tables 4 and 5). Correlating the short-form with the original 70-item version of the instrument, it became clear that there is strong overlap between the two (*r* ~ .90 and greater), and the original meanings of the JAS-70 subscales and the total have been retained. Nonetheless, there were some improvements in terms of its discriminant validity: The mean inter-correlations between its subscales went from *r* = .839 to *r* = .666. Despite the latter still being a highly significant correlation, it is considerably smaller than the mean overlap of the original, Δ*r* = .173, *z* = 14.07, *p* < .001. In terms of convergent validity, we found the expected pattern of correlations with the HEALTH-49. Namely, symptoms of mental distress and social restrictions correlated positively with job anxiety, and indicators of well-being and social integration evinced negative associations. To synthesize these results into a more comprehensive format we also ran a canonical correlation analysis. This yielded canonical correlation coefficients *R* of .571, .248, .218, .144, and .093 – with the first three being significant contributors (*p* < .001).

**Table 4:** Correlations within and between the JAS-15 and -70

	A^15^	B^15^	C^15^	D^15^	E^15^	Corr. Total^15^	A^70^	B^70^	C^70^	D^70^	E^70^	Corr. Total^70^
A^15^	–	.699	.704	.700	.629	.808	.910	.813	.760	.740	.677	.835
B^15^		–	.624	.621	.526	.705	.727	.887	.639	.645	.606	.711
C^15^			–	.803	.658	.823	.812	.720	.916	.791	.679	.825
D^15^				–	.699	.847	.846	.727	.873	.896	.699	.875
E^15^					–	.736	.739	.655	.713	.731	.879	.770
Corr. Total^15^						–	.915	.834	.880	.857	.767	–
A^70^							–	.852	.892	.860	.758	.931
B^70^								–	.759	.782	.731	.848
C^70^									–	.867	.730	.894
D^70^										–	.772	.899
E^70^											–	.805
Corr. Total^70^												–

^15^ = Scales of the shortened Job Anxiety Scale; ^70^ = Scales of the original Job Anxiety Scale; Corr. Total = The corrected scale total, excluding the respective subscale; A = Stimulus-related anxiety and avoidance behavior; B = Social anxiety and cognition of mobbing; C = Health- and body-related anxieties; D = Cognition of insufficiency; E = Job-related worrying; all correlations are significant at *p* < .001

**Table 5:** Correlations between the JAS-15 and the HEALTH-49

	A	B	C	D	E	Total
HEALTH Somatoform symptoms	.236^**^	.175^**^	.279^**^	.286^**^	.329^**^	.304^**^
HEALTH Depressive symptoms	.420^**^	.347^**^	.329^**^	.386^**^	.435^**^	.443^**^
HEALTH Phobic/Anxious symptoms	.434^**^	.282^**^	.290^**^	.347^**^	.364^**^	.397^**^
HEALTH Psychological and somatoform symptoms	.457^**^	.347^**^	.382^**^	.433^**^	.452^**^	.479^**^
HEALTH Psychological well-being	−.231^**^	−.209^**^	−.205^**^	−.248^**^	−.262^**^	−.267^**^
HEALTH Difficulties in interactions	.347^**^	.360^**^	.256^**^	.357^**^	.366^**^	.387^**^
HEALTH Self-efficacy	−.353^**^	−.268^**^	−.286^**^	−.345^**^	−.333^**^	−.367^**^
HEALTH Activity and participation	−.246^**^	−.220^**^	−.239^**^	−.277^**^	−.251^**^	−.286^**^
HEALTH Social support	−.145^**^	−.103^**^	−.093^*^	−.087^*^	−.078^*^	−.116^**^
HEALTH Social distress	.247^**^	.182^**^	.119^**^	.197^**^	.209^**^	.219^**^

JAS-15 = Shortened Job Anxiety Scale; HEALTH-49 = Hamburg Modules for the Assessment of Psychosocial Health; A = Stimulus-related anxiety and avoidance behavior; B = Social anxiety and cognition of mobbing; C = Health- and body-related anxieties; D = Cognition of insufficiency; E = Job-related worrying; ^**^ = Significant at *p* < .01; ^*^ = Significant at *p* < .05

## Discussion

The present study had two aims. The first one was to develop a new short scale of the JAS. The second aim was to evaluate the psychometric properties of this new JAS short scale. The initial goal might seem superfluous at first due to the existence of the Workplace Phobia Scale (WPS [18]). However, this scale focuses on stimulus related panic symptoms and avoidance behavior; that are the two typical aspects of phobias diagnoses. Therefore, it is a useful clinical tool to screen for work place phobia. In contrast, the new JAS short scale is an empirically-derived extract of items containing job related anxiety symptoms. It is thus based on a much wider construct – retaining all five dimensions that made up the original 70-item JAS. This goal was achieved by using model comparisons based on ant-colony optimization. As a result, a JAS short scale consisting of 15 items was created.

The second goal was to evaluate the psychometric properties of this new JAS short scale. In the present study, the JAS (70 items) was found to be highly reliable (ω = .98). This result accords well with the research conducted by Linden et al. [9] who found very good values for Cronbach’s alpha (α = .98) as well. The new short JAS scale (15 items) also achieves a very good level of reliability (ω =. 95). Even though the reliability drops from .98 to .95, it can nevertheless be interpreted as being a very high value. The level of reliability usually drops when the number of equally well-fitting items is reduced [35]. Apart from the JAS-15 being a reliable scale, we also found evidence for its strict measurement invariance across age groups and participant sex. This means that group means can be meaningfully compared and inferences can be drawn from these comparisons.

A strength of the present study and the JAS-15, is that we disentangled the JAS dimensions and thus lowered their average inter-correlation substantially. While the average correlation of *r* = .666 is still high, the subscales are not redundant as shown in factor analysis. In addition, we retained most of the JAS-15’s overall predictive power, as evidenced by a near-1-correlation between the JAS-15 and JAS-70 totals. Moreover, the JAS-15 and its subscales displayed convergent validity with a measure of psychosocial health in the expected manner. It should be noted that the JAS correlated roughly equally (*r* ~ .30 to .40) with the phobia/anxiety subscale of the instrument and with other measures of psychological distress. This apparent “lack” of differential correlation patterns between the different forms of psychological distress can be explained by the fact that the phobia/anxiety subscale of the HEALTH is focused on classic phobia symptoms such as agoraphobia and specific phobias (such as fear of elevators).

### Limitations

Since the JAS is a self-report scale the validity of the assessment is tied to the individuals responding to it. Among other works, Razavi [36] discusses the shortcomings of these measures – such as acquiescence and social desirability – as well as potential remedies.

The study is based on data collected in a clinical environment with a large proportion of psychosomatic and rehabilitation patients. Therefore, it appears questionable that the can be transferred without reservation to other clinical and nonclinical populations. Additionally, the sample consisted of 991 patients from two different clinics. A larger sample size from more clinics – or even from the general population – would provide an even wider database.

Only little research has been carried out concerning job-related anxiety. Usually, researchers adapt different instruments or constructs in order to measure job anxiety. Therefore, further research in clinical and nonclinical samples will be necessary in order to understand the underlying construct of job related anxiety. Based on this knowledge, the JAS should be subject to further testing and be further developed. Also, so far it is still unclear how sensitive the JAS might react to changes in a person or an organization. Therefore, the sensitivity of the JAS regarding changes should be tested.

## Conclusion

The aim of this study was to create a new, empirically derived version of the JAS that is both short and efficient and also to assess their psychometric properties. The new JAS short form consists of 15 items, retaining the original five dimensions. Thus, the JAS short form will be a helpful instrument in order to screen job related anxiety in an efficient manner.

## Data Availability

All data and materials are available from the corresponding author upon reasonable request.

## Abbreviations

JAS: Job Anxiety Scale
WPS: Workplace Phobia Scale
CFI: Comparative Fit Index
TLI: Tucker-Lewis Index
RMSEA: Root Mean Square Error of Approximation
SRMR: Standardized Root Mean Square Residual
GH: Gamma Hat
ICD: International Statistical Classification of Diseases and Related Health Problems
DSM: Diagnostic and Statistical Manual of Mental Disorders
STAI-T: Stait-Trait-Anxiety Inventory
HEALTH: Hamburg Modules for the Assessment of Psychosoical Health
